This article has been retracted.

# MiR-124 acts as a target for Alzheimer’s disease by regulating BACE1

**DOI:** 10.18632/oncotarget.23119

**Published:** 2017-12-09

**Authors:** Fengmao An, Guohua Gong, Yu Wang, Ming Bian, Lijun Yu, Chengxi Wei

**Affiliations:** ^1^ Medicinal Chemistry and Pharmacology Institute, Inner Mongolia University for The Nationalities, Tongliao, Inner Mongolia, P.R. China; ^2^ Inner Mongolia Key Laboratory of Mongolian Medicine Pharmacology for Cardio-Cerebral Vascular System, Tongliao, Inner Mongolia, P.R. China; ^3^ First Clinical Medical of Inner Mongolia University for Nationalities, Tongliao, Inner Mongolia, P.R. China

**Keywords:** Alzheimer’s disease, miR-124, BACE1, cell viability, cell apoptosis

## Abstract

Although large numbers of microRNAs (miRNAs) expressed in Alzheimer disease (AD) have been detected, their functions and mechanisms of regulation remain to be fully clarified. Beta-site Amyloid precursor protein Cleaving Enzyme 1 (BACE1) has been one of the prime therapeutic targets for AD. Here, we identified that miR-124 levels are gradually decreased in AD. In addition, we demonstrated that miR-124 suppresses BACE1 expression by directly targeting the 3′UTR of Bace1 mRNA *in vitro*. Inhibition of miR-124 significantly increased BACE1 levels in neuronal cells. In contrast, miR-124 overexpression significantly suppressed BACE1 expression in cells. And finally we determined that downregulation of miR-124 alleviated Aβ-induced viability inhibition and decreased apoptosis in SH-SY5Y cells. Our results demonstrated that miR-124 is a potent negative regulator of BACE1 in the cellular AD phenotype and might be involved in the pathogenesis of AD.

## INTRODUCTION

Alzheimer's disease (AD), as many researchers know, is the most common neurodegenerative diseases which has the characters of increasing dysfunction in mental behavior and progressive impairment of memory [1]. Abnormal upregulation of amyloid-β (Aβ) peptide is the major causes of AD [2]. Beta-site amyloid precursor protein cleaving enzyme 1 (BACE1) is the key enzyme which regulated the production of Aβ. Given its critical role in Aβ production, it has been possible that BACE1 could be act as a therapeutic target for AD and Alzheimer`s β-secretase [3].

MicroRNAs (miRs) are small non-coding RNAs that regulate a large number of gene expression [4, 5]. Altered miRNA expression is thought to be involved in various biological processes and pathological processes including AD [6-8]. The three precursor variants of miR-124 are located at the points of chromosomes 8p23.1, 8q12.3 and 20q13.33, respectively [9]. MiR-124 is a neurosystem-specific miRNA which play crucial roles in the nervous system [10, 11]. MiR-124 has multiple downstream targets and its aberrant expression is involved in the feedback loops of gene regulation networks [12, 13]. However, the expression and role of miR-124 have not been explored in AD development. The underlying mechanism remains unexplored. In this study, we examined the expression and biological function of miR-124 in AD. We also investigated its potential possible mechanism and found that miR-124 regulates AD progression through regulation of BACE1.

## RESULTS

To explore the role of miR-124 in the pathogenesis of AD, miR-124 expression was examined using qRT-PCR analysis in 35 cases of sporadic AD brain tissues and 35 cases of normal control subjects. MiR-124 expression was significantly reduced in AD brain tissues compared with the control group (*P* < 0.01; Figure 1A). To further quantify the expression level of BACE1, we detect the expression levels of BACE1 mRNA in sporadic AD tissues using qRT-PCR analysis. As shown in Figure 1B, AD samples showed elevated BACE1 expression (*P* < 0.01). There was a significantly higher level of BACE1 protein expression in sporadic AD brain samples compared with the normal samples (Figure 1C).

**Figure 1:** The relative expression of miR-124 and BACE1 were determined by qRT-PCR and western blot in AD patients **(A)** miR-124 expression levels were significantly lower in sporadic AD brain tissues than control tissues; **(B)** BACE mRNA expression levels were significantly higher in sporadic AD brain tissues than control tissues; **(C)** BACE1 protein expression levels were significantly higher in AD group than in control group.

In order to evaluate the effect of miR-124 on the Aβ-induced inhibition of cell growth, SH-SY5Y cells were transiently transfected with miR-124 inhibitors (anti-miR-124). Then we investigate the effect of inhibition of miR-124 on the cell viability of SH-SY5Y cells by MTT assay. We found that Aβ markedly suppressed SH-SY5Y cell viability, and inhibition of BACE1 could enhance this effect (Figure 2A). However, knockdown miR-124 alleviated the viability inhibition of SH-SY5Y cells by Aβ (Figure 2B).

**Figure 2:** **(A)** MTT assay results showed that Aβ inhibited the viability of SH-SY5Y cells and downregulation of BACE1 enhanced the inhibitory effects of Aβ; **(B)** downregulation of miR-124 relieved Aβ-induced viability inhibition of SH-SY5Y cells; **(C)** flow cytometric analysis results showed that Aβ-induced apoptosis of SH-SY5Y cells and downregulation of BACE1 enhanced the induced effects of Aβ; **(D)** downregulation of miR-124 decreased apoptosis of SH-SY5Y cells in the presence of Aβ.

We further investigated whether miR-124 regulates neuron survival by orchestrating apoptosis. The Flow cytometric analysis indicated apoptosis of SH-SY5Y cells was increased after treatment of Aβ. Knockdown of BACE1 could enhance the effects of Aβ, however, miR-124 inhibitor attenuated Aβ induced apoptosis in SH-SY5Y cells (Figure 2C and 2D); therefore, the present results suggest that miR-124 inhibited Aβ-induced cell proliferation and induced Aβ-induced apoptosis *in vitro*.

To demonstrate this conclusions further, potential target genes for miR-124 were therefore searched for using bioinformatics software. One potential miR-124 binding sites were located in the 3’ UTR of BACE1, indicating that BACE1 is one of the candidates (Figure 3A). To validate our hypothesis, the wild-type (WT) 3’UTR of BACE1 and its corresponding mutant (MUT) counterparts were clone into luciferase vector. Relative luciferase activity assays revealed that the luciferase intensity was suppressed by overexpresses of miR-124, but not in mutant 3’UTR (Figure 3B).

**Figure 3:** BACE1 is one of the candidates because miR-124 includes its potential binding sequences of the BACE1 mRNA 3′-UTR; miR-124 regulates BACE1 expression by directly binding to the 3′-UTR of BACE1 mRNA **(A)** The putative binding sites of miR-124 in the wild-type 3′-UTR of BACE1 (BACE1 3′-UTR-WT) and mutated target sites of BACE1 (BACE1 3′-UTR-MUT). **(B)** Relative luciferase activity in HEK293 cells co-transfected with pGL3-BACE1–3′-UTRWT/MUT and miR-124 mimics or miRNA scramble control (miRcon).

To further confirm that whether the BACE1 expression level is negative controlled by miR-124, we determined effects of miR-124 mimics or inhibitors on BACE1 in SH-SY5Y cells. The treatment of miR-124 mimics dramatically downregulated BACE1 mRNA and protein, and inhibition of miR-124 significantly increased the levels of BACE1 mRNA and protein (Figure 4A and 4B; either *P* < 0.05), suggesting that binding of miR-124 to BACE1 is important for blocking BACE1 expression.

**Figure 4:** The relative levels of BACE1 mRNA and protein in SH-SY5Y cells transfected with miR-124 mimics, miRNA mimic negative control (miR-con), miR-124 inhibitors (anti-miR-124), or miRNA inhibitor negative control (anti-miR-con) **(A)** At 48 h posttransfection, the relative levels of BACE1 mRNA were measured using qRT-PCR. **(B)** At 48 h posttransfection, the relative levels of BACE1 protein were measured using western blotting. Data are shown as means ± standard deviation (SD). ^**^P < 0.01.

## DISCUSSION

AD is a progressive neurodegenerative disease leading to deteriorating cognitive and memory function, immobility, and eventually death in affected patients [14]. The accumulation of Aβ and the formation of neurofibrillary tangles are considered as the main pathogenies of AD [15]. BACE1 plays an crucial role in the production of Aβ from AβPP [3]. Our observations suggest that miR-124 may be a negative regulator of BACE1 in AD and that expression of miR-124 might represent a further step towards the phenotype of AD.

Recently, increasing reports have indicated the importance of specific miRNAs in progression of various diseases; however, only a few reports have addressed the function of miRNAs in AD pathogenesis [16-18]. MiR-124, enriched in neurons, has been implicated as a mediator of nerve system [19]. Previous studies have suggested miR-124 alleviated the cell death in the process of AD [20]. Fang et al. reported that miR-124 is notably abnormal in AD by targeting with BACE1. MiR-124 was demonstrated to alter chromatin structure and regulate gene expression, thereby giving rise to a cell death phenotype. However, the mechanisms that regulated by miR-124`expression in AD are poorly defined.

We found that miR-124 was decreased in the AD tissues, and BACE1 was increased in the AD tissues, implying that miR-124 might be an useful therapeutic target in AD. We then attempt to identify novel mechanisms regulating BACE1 expression. Bioinformatics software identified that BACE1 is the target of miR-124. Luciferase reporter assays showed that upregulation of miR-124 resulted in a consistent attenuation of the expression of a luciferase reporter containing WT of BACE1. The miR-124 inhibitor against its target gene and miR-124 mimics were transfected into SH-SY5Y cells to modulate the BACE1 activity and thus determine the miR-124 affects cell phenotypes by the direct regulation of BACE1. Our discovery that miR-124 inhibits BACE1 activity and is commonly down-regulated in AD may provide a novel therapeutic avenue, as miRNA could potentially be used to modulate BACE1.

In summary, we found that miR-124 is an important modifier of development of AD which regulates the expression of BACE1 that contribute to pathogenesis of AD. These findings may not only increase our knowledge of AD development, but also help with therapeutic strategies for AD.

## MATERIALS AND METHODS

### Human brain tissue

35 AD patients and 35 control subjects were implicated in this study. Frozen tissue samples of frontal cortices from autopsied and histopathologically confirmed AD and control cases were obtained from the University General Hospital. Each tissue sample was homogenized to 10% (w/v) final concentration in ice-cold 1x phosphate buffer solution (PBS), supplemented with Ribonu-clease inhibitor (Takara, Tokyo, Japan) and protease inhibitor cocktail (Roche Diagnostics, GmbH, Germany). And each homogenized sample was used for cellular extraction for mRNA, miRNA and protein. Prior to the operation, patients granted consent for the use of the excised brain tissue in medical or scientific research. And the use of frozen human brain tissue was approved by the Institutional Review Board of University for the Nationalities.

### Cell culture and treatment

Human neuroblastoma SH-SY5Y cells and human embryonic kidney 293 cells (HEK293) were provided by the cell resource center of Chinese academy of medical sciences (Beijing, China). Cells were cultured in Dulbecco’s modified Eagle’s medium (DMEM) (Invitrogen, Carlsbad, CA, USA) containing 10 % heat-inactivated fetal bovine serum (FBS; Invitrogen), 100 units/ml penicillin, and 100 μg/mL of streptomycin (Sigma-Aldrich, St. Louis, USA) in a 37 °C and 5 % CO2 incubator. To obtain the neurotoxic form of Aβ, Aβ42 (Sigma-Aldrich) solution was keep at 37 °C for 4 days to induce an aggregated form of Aβ42 according to the methods described previously [7]. The aggregated form of Aβ42 was used at a final concentration of 10 μM. Twenty-four hours after transfection, SHSY5Y cells were subjected to Aβ treatment for 24 h. Cell viability and apoptosis were determined using 3-(4,5-dimethylthiazol-2-yl)-2,5-diphenyltetrazolium bromide (MTT) assay and flow cytometric analysis, respectively.

### Transfection

MiR-124 mimics, miRNA mimic negative control (miRcon), miR-124 inhibitors (anti-miR-124), and miRNA inhibitor negative control (anti-miR-con) were purchased from GenePharma (Shanghai, China). Synthetic miR-124 mimics, miR-con, miR-124 inhibitors, and anti-miR-con were transfected into cells using Lipofectamine 2000 (Invitrogen) according to the manufacturer’s instructions. Small interfering RNA (siRNA) vectors targeting BACE1 were purchased from GenePharma (Shanghai, China). Transfection was conducted using Lipofectamine 2000 (Invitrogen) according to manufacturer’s instructions.

### Quantitative real-time PCR

Total RNA and miRNAs were isolated using Trizol reagent (Invitrogen) and mirVana miRNA isolation kit (Ambion, Austin, TX, USA). Then cDNA was obtained by using oligo-dT primers or stem-loop reverse transcriptase (RT) primers, respectively. β-actin and U6 were used as controls for BACE1 and miR-124, respectively. PCR was performed under the following conditions: 94°C for 4 min followed by 40 cycles at 94°C for 1 min, 56°C for 1 min and 72°C for 1 min. Relative expression levels of the genes were calculated using the 2^-ΔΔCt^ method.

### Western blot assay

At the indicated times (at 48 h after transfection), cells were harvested in ice-cold PBS and lysates were prepared by RIPA buffer (Beyotime, China). Protein concentration was determined by BCA Protein Assay Kit (Beyotime, China) at 570 nm. Equal amounts of protein were separated by 8% or 15% SDS–PAGE gels. Then gels were transferred onto polyvinylidene fluoride (PVDF) membranes (Millipore, Billerica, MS, USA). Furthermore, for immunoblot experiments, the membranes were blocked for 2 h with 5% nonfat milk in Tris-buffered saline containing 0.1% Tween-20 (TBST) and were incubated with primary antibodies against BACE1 (Cat# ab2077,1:200, Abcam, Cambridge, MA) at 4°C for overnight, and then incubated with HRP-conjugated secondary anti-mouse or anti-rabbit antibodies (Multi Sciences, China) for 1 h at room temperature after washing. At last, membranes were visualized by a commercial enhanced chemiluminescent substrate (Bio-Rad, USA), and Image J was used to quantitate the expression of proteins.

### Luciferase reporting assay

The 3’ UTR of BACE1 and the CMV promoter were amplified from human chromosomal DNA and pcDNA3.1 (+) and cloned into the pGL3-luciferase basic vector (Promega, Madison, WI, USA). Sequences of primers and cloning strategy are available on request. For the luciferase assays, 50 nM of miR-16b mimics or scrambled RNA were co-transfected with the reporter vector and the Renilla control vector (Promega, Madison, WI, USA) into the HEK293 cells by Lipofectamine 2000 (Invitrogen, Carlsbad, CA, USA). 24 h post transfection, the measurements were performed using the Dual luciferase re-porter assay kit (Promega, Madison, WI, USA). Or the HEK293 cells post the transfection for 24 h was lyzed for western blot analysis.

### Determination of cell proliferation

Forty-eight hours after transfection, 3000 cells per well were seeded into 96-well plates. After 6, 24, 48, 72 and 96 h of culture, cell viability was measured using the Cell Proliferation Reagent Kit I (MTT; Roche Applied Science).

### Flow cytometric analysis

Cells were harvested directly or 48 h after siRNA transient transfection and washed with ice-cold phosphate-buffered saline (PBS). The annexin V-fluorescein isothiocyanate (FITC) apoptosis detection kits (KeyGEN Biotech, Nanjing, China) was used to detect apoptosis in a FACScan instrument (Becton Dickinson,, Mountain View, CA, USA), respectively.

### Statistical evaluation

Each experiment was performed as least three times and the data are expressed as the mean ± standard error. For the analysis of miR-124 and U6, BACE1 and β-actin in mRNA or in protein level in protein level, between two groups, and data were analyzed using the Student’s t test. The nonparametric Pearson’s correlation test was performed to evaluate the correlation of miR-124 with the BACE1 mRNA level. A statistical significance was considered when *P* < 0.05. *P*<0.05 was considered to indicate a statistically significant difference. All statistical analyses were performed using the SPSS 10.0 statistical software package (SPSS, Inc., Chicago, IL, USA).
